The article "Research on Virtual Interactive Animation Design System Based on Deep Learning" was retracted in 2023. Reasons: unreliable results or conclusions; concerns about the data; concerns about the results or conclusions; concerns about the peer review.

# Research on Virtual Interactive Animation Design System Based on Deep Learning

**DOI:** 10.1155/2022/5035369

**Published:** 2022-06-25

**Authors:** Bing Liu

**Affiliations:** JMU College of Arts & Design, Xiamen 361000, China

## Abstract

With the rapid development of computer network technology, the advantages of virtual reality technology in the field of instant messaging are becoming more and more significant. Virtual reality technology plays an important role in communication networks, including enhanced resource utilization, device redundancy, immersion, interactivity, conceptualization, and holography. In this paper, we use the basic theory of Restricted Boltzmann Machine to establish a semisupervised spatio-temporal feature model through the animation capture data style recognition problem. The bottom layer can be pretrained with a large amount of unlabeled data to enhance the model's feature perception capability of animation data, and then train the high-level supervised model with the labeled data to finally obtain the model parameters that can be used for the recognition task. The layer-by-layer training method makes the model have good parallelism, that is, when the layer-by-layer training method makes the model well parallelized, that is, when the bottom features cannot effectively represent the animation features, such as overfitting or underfitting, only the bottom model needs to be retrained, while the top model parameters can be kept unchanged. Simulation experiments show that the design assistance time of this paper's scheme for animation is reduced by 10 minutes compared to baseline.

## 1. Introduction

Video communication in instant messaging systems usually requires high real time and stability; otherwise, it is prone to data delay, playback lag, and other instability [1]. Due to the influence of unstable network environment, the data is easily disturbed by various factors during transmission, resulting in the data not being broadcasted properly at the receiving end [2]. And the goal of this paper is to design a virtual video chat system combined with virtual reality, which needs to transform from the original transmission video data to the transmission user's face key point data based on the application scenario and handle the transmission abnormality [3]. At the same time, because the content of this paper is not based on video streaming instant messaging, but 3D virtual animation video chat, the user sees the expression animation of the virtual animation model during the chat, so the data format transmitted in the network is the data set of face keypoints and voice data, and this paper has high requirements for noise reduction and echo cancellation of voice based on the actual application scenario, thus making the voice and animation [4]. Therefore, the synchronization of voice and animation and speech optimization become the urgent problem in the subject.

The article "Research on Virtual Interactive Animation Design System Based on Deep Learning" was retracted in 2023. Reasons: unreliable results or conclusions; concerns about the data; concerns about the results or conclusions; concerns about the peer review.

In recent years, the research on face keypoint localization has become more and more abundant and mature, and the research on deep learning has also made many breakthroughs, bringing better innovative methods and more opportunities for other related research fields [5]. Face keypoint localization is the basis of face recognition and other research, and the application scenarios are very broad. Researchers have proposed many algorithms for face keypoint localization and achieved good results in related fields, but in practical applications, faces are often affected by various internal and external factors such as expression, posture, illumination, and occlusion, making it very difficult to achieve accurate face keypoint localization, which is still a great challenge [6, 7]. This paper will address the design and optimization of the face keypoint localization model and its application in mobile based on practical application scenarios [8].

Virtual reality technology is an important part of the computer field and has important applications in biochemistry, social entertainment, aerospace, and military industries [9]. However, virtual reality technology is less present in the current popular instant messaging-related research, which indicates that researchers in the field of instant messaging have paid less attention to virtual reality technology and have not well combined the two [10]. In this paper, we combine virtual reality technology and instant messaging, and the client drives the expression animation of 3D virtual model by parsing the key point data of human face to realize the virtual animation real-time communication [11].

In summary, the design of combining virtual reality technology with instant messaging and combining human-computer interaction with video chat will be a very important research direction in the future communication field [12].

## 2. Related Work

At present, domestic and foreign research in instant communication has made great progress, and communication among people has become more and more convenient and colorful [13]. At the same time, people are more and more willing to try various diversified and personalized instant communication methods, such as using 3D virtual animation models instead of real faces to communicate in real time, and the expression animation of 3D virtual animation models is driven by the real expressions of users in real time [14, 15].

In this paper, we combine deep machine learning-based face keypoint localization technology, virtual reality technology, and instant messaging to design and implement a more personalized instant messaging system [16].

The article "Research on Virtual Interactive Animation Design System Based on Deep Learning" was retracted in 2023. Reasons: unreliable results or conclusions; concerns about the data; concerns about the results or conclusions; concerns about the peer review.

### 2.1. Face Key Points

Face keypoint localization is the basis of face recognition and expression analysis and has a very broad development and application prospect. Researchers have proposed many face keypoint localization algorithms based on various methods. In [17], a fast face alignment method based on a layer-by-layer model is proposed, which converges after 8∼10 iterations and the alignment time of each face image is tested within 40 ms on a Samsung I9300 smartphone. Reference [18] proposed a multitask cascaded convolutional neural network to achieve face detection while achieving face key point localization. Reference [12] et al. used a cascaded convolutional neural network-based method to achieve the localization of five key points of faces with an average localization error of 1.264 pixels, and it only takes 15.9 ms to process a face image. Reference [19] proposed a new cascaded deep design warp network, where the input of the previous cascaded neural network is a certain part of the image, unlike the previous ones, the input of each stage of the DAN (Deep Alignment Network) network is the whole image, which can extract features from the whole image. The features can be extracted from the whole image to obtain more accurate localization. Reference [20] proposed an edge-aware face alignment algorithm based on the edge as the geometric structure of the face for localization of 98 key points of the face.

From the above studies, it can be seen that there are abundant studies on face keypoint localization techniques and many algorithms are able to achieve better results. In the task of this paper, we are more concerned with the real time of face keypoint localization and the accuracy of face keypoint localization under different postures and expressions.

### 2.2. Data Transmission and Sound-Image Synchronization

Currently, data transmission is moving in two directions: first, to pursue higher transmission performance at lower transmission rates, that is, to reduce the transmission BER as much as possible; second, to increase the transmission rate as much as possible while the BER meets the requirements. Reference [11] proposes a new method for synchronizing audio and video presynchronization: by designing a presynchronization module based on the RTP/RTCP timestamp in the receive buffer and a new working mechanism, a fast synchronization within the media is achieved, eliminating the intermediate layer bias and adding no additional end-to-end delay before unpacking the RTP packets. Reference [12] proposes a method that uses timestamps to store audio and video data with correlation in acquisition time into a fixed synchronization data structure and always synchronize and control them during acquisition, encoding, transmission, reception, decoding, and playback, which can well meet the demand of audio and video synchronization in application scenarios and has good engineering practice. Reference [15] implemented a virtual reality-based gaze sensitive social communication system for autistic patients, which can measure the gaze-related index of patients during their interaction with virtual companions, and this index can be mapped to their corresponding anxiety level. At the same time, the system can influence the patient's task performance and gaze-related index in response to the virtual companion's emotions.

The article "Research on Virtual Interactive Animation Design System Based on Deep Learning" was retracted in 2023. Reasons: unreliable results or conclusions; concerns about the data; concerns about the results or conclusions; concerns about the peer review.

Technologies such as speech coding and decoding, data transmission, and audio and video synchronization are the basis of research in instant messaging. In the task of this paper, more attention is paid to the effect of special environment on speech, such as external playback under mobile devices and the synchronization of speech with 3D animation models.

## 3. Animation Design Model Based on Two-Layer RBM

Aiming at the problem that there is often a semantic gap between the underlying features and the high-level semantics of animation capture data, a semantic recognition algorithm for animation capture data that incorporates a restricted Boltzmann machine generative model and a discriminative model is proposed by combining deep learning ideas. The algorithm adopts a two-layer restricted Boltzmann machine to perform discriminative feature extraction (feature extraction layer) and style recognition (semantic discriminative layer) on animation capture data, respectively. Firstly, considering that the autoregressive model has excellent ability to express temporal information, a conditional restricted Boltzmann machine generative model based on single-channel ternary factor interaction is constructed for extracting temporal feature information of animation capture data; then, the extracted features are then coupled with the corresponding style labels as the input of the current frame data layer of the restricted Boltzmann machine discriminative model in the semantic discriminative layer for the training of single-frame style recognition; finally, on the basis of obtaining the parameters of each frame, the voting space is added to the top of the model to achieve the effective recognition of the style semantics of the animation capture sequence. The experimental results show that the algorithm has good robustness and scalability, can meet the needs of diverse animation sequence recognition, and facilitate the effective reuse of data.

The article "Research on Virtual Interactive Animation Design System Based on Deep Learning" was retracted in 2023. Reasons: unreliable results or conclusions; concerns about the data; concerns about the results or conclusions; concerns about the peer review.

### 3.1. Introduction to Recognition Models and Processes

As one of the representative models of deep learning, the RBM model has the ability to extract static frame features and build a CRBM model by adding autoregressive model constraints to the input layer, which in turn can obtain temporal feature information with contextual semantic scenarios. Reference [19] proposes a nonlinear mapping threshold CRBM binary hidden variable probabilistic model, which uses an unsupervised learning algorithm to extract not only the highly structured feature information that is available when transitions are transferred between video frame images, but also to portray the spatial relationships between each frame's own pixels. In this paper, a voting space layer is added on top of the label layer for animation design, and a segmentation layer with the ability to identify transition frames can also be added. The animation design process using the two-layer RBM model is shown in Figure 1.

### 3.2. Bottom Feature Extraction Layer

The generative model fully considers the distribution of data and can use joint probability to get the conditional probability from input data to output data. Therefore, the RBM based on the generative model can reflect the generation process of the target object and the similarity between similar objects through the energy function and the activation state of the hidden layer neurons. The layer 1 generative RBM model developed in this paper takes advantage of the second property.

According to the autoregressive model algorithm, this paper splits the animation into 2 parts and constructs the bottom spatio-temporal feature layer: one part represents the previous *n* frames of the current animation frame, which is called the history frame; the other part has only one frame, which represents the current animation frame, which is called the current frame. In addition, the interaction factor layer is added to realize the information interaction control between the 2 input layers and the feature layer, aiming to map the latent information and spatio-temporal feature information in the animation data to the feature representation layer through the factor layer so as to obtain more accurate probability distribution of the data in the process of reverse estimation; meanwhile, the factor layer also has the function of reducing the model space complexity from *o*(*n*^3^) to *o*(*n*^2^), which is described as follows.

The representation of each neuron in the history frame based on the RBM feature learning is *p*=(*p*_1_, *p*_2_, ..., *p*_*m*_), where *m*=(*f*_*r*_ − 1)*d* is the total number of neurons, *f*_*r*_ denotes the length of the historical frame, and *d* denotes the frame data dimension. The neurons of the current frame are represented as *n* = *d*, with*v*=(*v*_1_, *v*_2_, ..., *v*_*n*_) representing the total number of neurons of the current frame. The hidden layer neurons are represented as *h*=(*h*_1_, *h*_2_, ..., *h*_*t*_) , where *t* is the total number of hidden layer neurons set. For the convenience of description, *p*_*i*_ is the *i*th neuron of the history frame, *v*_*j*_ is the *j*th neuron of the current frame, *b*_*j*_ represents the bias of the *j*th neuron, *h*_*k*_ represents the *k*th neuron of the hidden layer, and *c*_*k*_ represents the bias of the *k*th neuron. *c*_*k*_ is the connection weight from the interaction factor layer to the history frame (directed connection), *W*_*if*_^*p*^ is the connection weight from the interaction factor layer to the current frame (directed connection), and *W*_*if*_^*v*^ is the connection weight from the interaction factor layer to the hidden layer (undirected connection). *W*_*kf*_^*H*^ is the connection weight from the interaction factor layer to the hidden layer (undirected connection), which determines the model parameters and is denoted as *θ*_1_=(*W*_*if*_^*P*^, *W*_*jf*_^*V*^, *W*_*kf*_^*H*^, *b*, *c*). Note that the history frame and the current frame are both real-parameter visible neurons, while the hidden layer is a binary random hidden unit.

The article "Research on Virtual Interactive Animation Design System Based on Deep Learning" was retracted in 2023. Reasons: unreliable results or conclusions; concerns about the data; concerns about the results or conclusions; concerns about the peer review.

### 3.3. High-Level Semantic Discriminant Layer

The DRBM model can be considered as a two-layer model, where both the visible layer and the label layer are the input sample data, and the hidden layer can be used to sample the joint probability distribution and conditional probability distribution of the visible and label layer data. Since an animation belongs to only one style, the label layer can be coded as “single heat”; that is, the label layer is set as a binary neuron, and only the neuron corresponding to the label has a value of 1 and is active [21, 22].

The parameters are defined as follows: the label layer neuron is *L*(*L*_1_, *L*_2_,…, *L*_0_), where *o* represents the number of all styles of training samples, and the bias is *T*=(*t*_1_, *t*_2_,…*t*_0_); the visible layer is the feature information extracted from the first layer, which is a real unit, denoted as *X*=(*x*_1_, *x*_2_,…*x*_*k*_), and the bias is *Q*=(*q*_1_, *q*_2_,…*q*_*k*_); the hidden layer is the unit that can represent the correspondence between the label layer and the visible layer, denoted as *Y*=(*y*_1_, *y*_2_,…*y*_*n*_), and the bias is *R*=(*r*_1_, *r*_2_,…*y*_*n*_). The connection weights of the visible and labeled layers to the hidden layer are *W*_*yx*_, *W*_*yl*_. Since this layer is used for classification rather than prediction of the probability distribution of the animated features, a hybrid discriminant method is used to train the second layer of the RBM, which is a linear combination of the optimal discriminant model *p*(*l|x*) and the generative model *p*(*l*, *x*). The training algorithm is still a comparative scattering algorithm. The log-likelihood function of the function to be optimized takes the form

(1) $$\begin{array}{c} L_{\theta_{2}}=\sum_{i=1}^{s}\log P\left(l_{i}|x_{i}\right)-\alpha \sum_{i=1}^{s}\log P\left(l_{i},x_{i}\right), \end{array}$$

where *s* denotes the total number of categories. For the 2nd term, i.e., the generative model part, the parameters are updated according to the steps of the 1st level [23, 24]. For the first discriminant model, the conditional distribution can be calculated as proposed by Larochelle et al.

(2) $$\begin{array}{c} P\left(l|x\right)=\frac{{\text{e}}^{\left(t_{l}+\Sigma_{j}\left(\log\;1+{\text{e}}^{i}W_{ji}x_{i}+W_{jl}+r_{j}\right)\right)}}{\sum_{ls}{\text{e}}^{\left(t_{ls}+\Sigma_{j}\log\left(1+{\text{e}}^{i}\right)\right)}}. \end{array}$$

In a sequence of frames, equation (3) represents the magnitude of the probability that each frame belongs to each label, where *l* is the category label notation to which the training frame belongs, *ls* ∈ (1,2,…, 0). Therefore, the conditional probability *p*(*l|x*) can be solved by an optimization function using the gradient descent method such that the probability that the animation feature *x* belongs to the correct label *l* is maximized. Then, for a single frame of animation *x*^(*t*)^ and the corresponding style label *l*^(*t*)^, there are

(3) $$\begin{array}{c} \frac{\partial \;\log P\left(l^{\left(t\right)}|x^{\left(t\right)}\right)}{\partial \theta_{2}}=\sum_{j}\mathrm{sigmod}\left(S\left(x^{\left(t\right)}\right)\right)\frac{\partial S\left(x^{\left(t\right)}\right)}{\partial \theta_{2}}-\sum_{j,ls}\mathrm{sigmod}\left(S\left(x\right)\right)P\left(ls|x^{\left(t\right)}\right)\frac{\partial S\left(x\right)}{\partial \theta_{2}}. \end{array}$$

Among them, *S*(*x*)=∑_*i*=1_^*k*^*W*_*ji*_*x*_*i*_+*U*_*jl*_+*r*_*j*_, *x*^(*t*)^ ∈ *x*. For label layer, bias update method is

(4) $$\begin{array}{c} \frac{\partial \;\log P\left(l^{\left(t\right)}|x^{\left(t\right)}\right)}{\partial t}=1_{y=y^{\left(t\right)}}-P\left(l|x^{\left(t\right)}\right), \end{array}$$

where 1_*y*_=*y*^(*t*)^ is the label layer neuron activated by the current label after the “single heat” encoding. The model parameters can be updated iteratively at each step by bringing equation (4) into the expression of the hybrid discriminative model in equation (3). The final DRBM model with classification function at layer 2 is trained [25, 26].

The article "Research on Virtual Interactive Animation Design System Based on Deep Learning" was retracted in 2023. Reasons: unreliable results or conclusions; concerns about the data; concerns about the results or conclusions; concerns about the peer review.

## 4. Experiment and Result Analysis

In order to verify the effectiveness of the two-layer model in animation design, the experiments are conducted on a PC with 3.30 GHz CPU and 8G memory, and the programming test environment is python3.7. In the generated model, the number of neurons in the historical and current frames as input data in the CRBM model is directly determined by the dimensionality of the input data. In the preprocessing, 53 dimensions of data were extracted for each frame, including 48 joint angular degrees of freedom, 3 animation directions, and 2 geodesic velocity data. The first 25 frames are used as the input vector of the history frame, and the 26th frame is used as the input data of the current frame so that the number of neurons of the history frame is 1325 and the number of neurons of the current frame is 53. The number of iterative updates is 250–500, and good feature information can be extracted.

### 4.1. Two-Layer Model Training

In this paper, we first eliminate the influence of spatial location of animation nodes on recognition and then retain the advantage of autoregressive model to build the first layer of ternary factor CRBM to extract temporal features and finally use the second layer of discriminative Boltzmann machine for classification. The two-layer model is trained to obtain a set of model parameters, including weights and biases, for each layer.

Since the layer 1 RBM uses a generative model, it contains reconstruction errors for the current frame animation data description. Using the reconstruction error, we can roughly determine how well the model fits the current 26-frame data distribution. If the error is too large, the parameters are not set properly and the number of neurons in the feature layer needs to be increased or the number of training sessions needs to be increased. Of course, the reconstruction error should not be too small, as overfitting will occur if it is too small. In the later tuning process, the appropriate number of hidden neurons and other techniques can reduce the occurrence of overfitting. In general, the reconstruction error will be stabilized within a certain range after a certain number of training sessions, which is verified by relevant experiments.

Figure 2 shows the reconstruction errors of layer 1 of the model for the 2 data sets. It can be seen that the reconstruction error obtained from the RBM model based on layer 1 will gradually stabilize after a certain number of iterations. For example, after 200 iterations, the reconstruction error basically tends to a stable level, and the total error of 53 Euler angles per frame does not exceed 0.9. Therefore, it can be judged that the layer 1 model does not change the original characteristics of the animation, and the fitting effect is relatively good.

The article "Research on Virtual Interactive Animation Design System Based on Deep Learning" was retracted in 2023. Reasons: unreliable results or conclusions; concerns about the data; concerns about the results or conclusions; concerns about the peer review.

To verify the reconstruction effect of the model on the animation style, Figure 3 shows the reconstructed effect of the 1st layer generating model part on the 4 end effectors (left and right hands, left and right feet) of the 1st animation style JO (jogging) of data set 1. Analyzing the fluctuation magnitude, we can see that the degree of change of the reconstructed data is similar to that of the original data animation style, which indicates that the data obtained by reconstructing using the first 25 frames and the model parameters are consistent with the style type of the current animation; that is, the hidden layer can effectively portray the style characteristics of the current animation.

The second semantic discriminative layer uses the RBM discriminative model to construct the mapping relationship between labels and each style animation feature, and the model parameters are updated according to the reconstruction errors of the input data in the label and feature layers. At the same time, a small number of samples are extracted from the training samples as the validation set to verify the accuracy of the model classification in each training cycle.  Figure 4 shows the variation of the free energy of the RBM model at layer 2 and the recognition rate of the validation set in Dataset 1 and Dataset 2 as the number of training cycles increases. The free energy is closely related to the probability distribution of the model, and the trend is inversely proportional to the change in the probability distribution, as the energy decreases, the probability distribution becomes closer to the feature distribution, which also validates the theory that the system is most stable at the lowest energy. The effect of model energy release on the recognition rate can be clearly observed in Figure 4(b): as the system stabilizes, the frame classification error of the validation set is in a decreasing state and gradually tends to be smooth.

### 4.2. Comparison and Analysis of Experimental Results

In order to further verify the recognition effect of the two-layer RBM model on animation style, the recognition results of this paper's algorithm are compared with the Adaptive Motion Codebook Classifier (AMCC) algorithm of [12] and the SVM recognition algorithm based on radial basis function, and the spatial locations of 23 nodes are selected as the data preprocessing method. The spatial position information of 23 nodes was selected as the data preprocessing method. From the experimental results of the three recognition algorithms in Figure 5, it can be seen that for simple animations, the two-layer RBM algorithm can also achieve good style determination results, such as JO, KF, and KS simple sequences, and its test discrimination rate reaches 100%. The main reason is that the AMCC and SVM algorithms mainly consider the spatial information of the body joints, which has the greatest influence on the animation style, for classification, and ignore the timing information. The two-layer RBM algorithm proposed in this paper can achieve better semantic discriminative effect, mainly because the first layer extracts discriminative spatio-temporal features for effective pose portrayal; the second layer of DRBM model can effectively sample the conditional probability distribution of feature layer and class label data for semantic discriminative effect.

The article "Research on Virtual Interactive Animation Design System Based on Deep Learning" was retracted in 2023. Reasons: unreliable results or conclusions; concerns about the data; concerns about the results or conclusions; concerns about the peer review.

In terms of space storage efficiency, the AMCC algorithm needs to store the entire training set and build codeword templates for different classes of animation sequences, so the space occupation rate is large. In contrast, the depth model built in this paper only needs 2 sets of finite parameters (1 set for each layer) to represent the sequence pose, and only some training samples are needed to learn the model parameters, so the storage space is relatively small. Therefore, the algorithm in this paper is suitable for the learning and modeling work of large data volume animation sequences. In terms of time efficiency, although the deep learning model established in this paper takes some time to learn the underlying features, once trained, the corresponding hidden units can be activated directly according to the model parameters and visible layer data, and the feature distribution of the current animation style can be obtained effectively. Therefore, the algorithm in this paper does not require additional similarity calculation, and in the MATLAB simulation environment, although the training time is long for 13 styles of animation, the recognition time is only 2.6 s. The speed of style recognition is comparable with existing algorithms, as shown in Figure 6.

## 5. Interactive Animation Design

In interactive animation design, the meaning of fast and slow rhythm is mostly reflected in the process of interactive experience. A fast rhythm can give immediate feedback to younger children. When children select options through the interactive buttons, as shown in Figure 7, the interactive buttons should change color and play corresponding music in an instant; for example, the button turns green with a celebratory tone when correct, and the mobile device vibrates and the button turns red when wrong. The immediate error feedback will provide a kind of error warning to the younger children so that they can form a psychological gap and pay attention to the subsequent case explanation.

The article "Research on Virtual Interactive Animation Design System Based on Deep Learning" was retracted in 2023. Reasons: unreliable results or conclusions; concerns about the data; concerns about the results or conclusions; concerns about the peer review.

From Figure 8, it can be seen that Dynamic algorithm and this paper's algorithm each have advantages in different styles of animation design. Dyneme vector-based recognition algorithm is weaker in the four animation styles of jump, lie, sit, and stand, because the algorithm does not sufficiently consider the backward and forward timing relationship, such as sitting on the ground and standing up from the ground are inverse animations, but their forward difference vectors are similar to each other. The algorithm in this paper overcomes this drawback by using the past frame cell layer and the current frame cell layer in the visible layer, but the shortcoming is that RBM has transfer invariance, which leads to interference in recognizing animation styles like deposit (picking something up from the ground), jog (running in place), rotate (rotating both arms), and so on, where the animation joint changes are similar but the joint positions are different. Interactive animation design should also anticipate in advance, using the platform's error record to analyze the error-prone content of younger children and insert.

## 6. Conclusion

In order to meet the demand for spatio-temporal feature representation in human animation design, this paper adopts the two-layer RBM algorithm for animation feature representation and style recognition. The experimental results show that RBM has very good advantages in feature extraction and can extract more discriminative spatio-temporal features of animation sequences after adding autoregressive model constraints; meanwhile, it can achieve very good style recognition effect after introducing Boltzmann machine discriminative model, but the algorithm also has certain shortcomings, mainly because the number of neurons of its deep learning model is difficult to be determined well. Animators can create a moderate risky situation in the interactive animation design. Young children are under the care and attention of parents and lack of emotional catharsis, which leads them to subconsciously like to take risks. Therefore, moderate increase of adventure elements can stimulate their interest and let their playful emotional needs be satisfied put.

## Figures and Tables

**Figure 1:** Flowchart of animation design based on two-layer RBM model.

**Figure 2:** Total error of RBM reconstruction in layer 1 versus the number of iterations. (a) Dataset 1. (b) Dataset 2.

The article "Research on Virtual Interactive Animation Design System Based on Deep Learning" was retracted in 2023. Reasons: unreliable results or conclusions; concerns about the data; concerns about the results or conclusions; concerns about the peer review.

**Figure 3:** Effect of end effector reconstruction. (a) Left foot. (b) Right foot. (c) Left hand. (d) Right hand.

**Figure 4:** Validation set error and energy change for 2 data sets. (a) Validation set error 1. (b) Free energy 1. (c) Validation set error 2. (d) Free energy 2.

**Figure 5:** Animation style recognition confusion matrix.

**Figure 6:** Comparison of animation design rates.

**Figure 7:** Animation design process.

**Figure 8:** Animated character design.

## Data Availability

The experimental data used to support the findings of this study are available from the corresponding author upon request.
